# Research on Chest Disease Recognition Based on Deep Hierarchical Learning Algorithm

This article has been retracted.

**DOI:** 10.1155/2022/6996444

**Published:** 2022-01-07

**Authors:** Lingling Li, Yangyang Long, Bangtong Huang, Zihong Chen, Zheng Liu, Zekun Yang

**Affiliations:** ^1^Department of Central Laboratory, Children's Hospital of Shanghai Jiao Tong University, Shanghai, China; ^2^School of Computing and Information System, University of Melbourne, Melbourne, Australia; ^3^School of Management, Shanghai University of Engineering Science, Shanghai, China; ^4^College of Engineering, Shantou University, Shantou, China; ^5^Department of Computer Science and Engineering, The Chinese University of Hong Kong, Shatin, Hong Kong, China

## Abstract

Chest X-ray has become one of the most common ways in diagnostic radiology exams, and this technology assists expert radiologists with finding the patients at potential risk of cardiopathy and lung diseases. However, it is still a challenge for expert radiologists to assess thousands of cases in a short period so that deep learning methods are introduced to tackle this problem. Since the diseases have correlations with each other and have hierarchical features, the traditional classification scheme could not achieve a good performance. In order to extract the correlation features among the diseases, some GCN-based models are introduced to combine the features extracted from the images to make prediction. This scheme can work well with the high quality of image features, so backbone with high computation cost plays a vital role in this scheme. However, a fast prediction in diagnostic radiology is also needed especially in case of emergency or region with low computation facilities, so we proposed an efficient convolutional neural network with GCN, which is named SGGCN, to meet the need of efficient computation and considerable accuracy. SGGCN used SGNet-101 as backbone, which is built by ShuffleGhost Block (Huang et al., 2021) to extract features with a low computation cost. In order to make sufficient usage of the information in GCN, a new GCN architecture is designed to combine information from different layers together in GCNM module so that we can utilize various hierarchical features and meanwhile make the GCN scheme faster. The experiment on CheXPert datasets illustrated that SGGCN achieves a considerable performance. Compared with GCN and ResNet-101 (He et al., 2015) backbone (test AUC 0.8080, parameters 4.7M and FLOPs 16.0B), the SGGCN achieves 0.7831 (−3.08%) test AUC with parameters 1.2M (−73.73%) and FLOPs 3.1B (−80.82%), where GCN with MobileNet (Sandler and Howard, 2018) backbone achieves 0.7531 (−6.79%) test AUC with parameters 0.5M (−88.46%) and FLOPs 0.66B (−95.88%).

## 1. Introduction

A potential risk of cardiopathy and lung disease threatens millions of lives, and most of these diseases are preventable due to the chest X-ray (CXR) technology. Now, CXR technology becomes a regular examination of heart and lung disease, which assists in clinical diagnosis and treatment. Some algorithms like convolutional neural network (CNN) and Bayesian models are introduced to process and make diseases prediction by CXR images, and they really make a difference. On the one hand, they reduce the workload of expert radiologists with the high speed of computation and make it possible for expert radiologists to process a huge number of radiology samples. On the other hand, these algorithms can filter out some low-risk radiology samples with a considerably low-false-negative rate so that expert radiologists can more easily find out the samples with potential risk.

CNN-based models can extract the features from images and use a fully connected layers to make prediction. Comparing to multi-class image classification [1], the multilabel task is more challenging due to the combinatorial nature of the output space. With the advent of deep learning, a more recent focus has been on adapting deep networks, typically convolutional neural networks (CNNs), for hierarchical classification [2, 3]. ResNet [4] was proposed to extract features with a deep convolutional network and improved the accuracy of ImageNet classification task. And now, ResNet is wildly used as a backbone to extract features, as well as pretrained model is adopted to accelerate the training procedure. But chest disease recognition task is a multilabel classification task, and the label (diseases) has hierarchical features, so the trick in classical image classification task might not work, if the hierarchical features are not properly extracted. Given the outstanding performance, deep learning has been applied in some safety and security critical tasks, such as self-driving, malware detection, identification [5], and anomaly detection [6].

In some previous work, Graph Convolution Network (GCN) [7] is introduced to learn the hierarchical features among the labels, and this kind of structure might be suitable for this chest disease recognition task. And works like MLGCN [8] designed a proper structure, utilized the hierarchical features of labels, and achieved a better performance, but most of them adopt a deep neural network like ResNet-101 as backbone to extract image features, which would suffer high cost of computation. In this work, we focus on the efficient computation in GCN. In order to decrease the parameters and FLOPs, firstly we designed a new backbone named SGNet-101, which is built by ShuffleGhost [9] block. The SGNet-101 utilized the redundancy of feature map in convolution and used ghost convolution to simulate the convolution scheme. Compared with light models which have wide usage of depthwise and elementwise convolution, SGNet-101 could reduce the FLOPs and parameters and maintain the image features more easily. In order to make sufficient usage of the information in GCN, we designed a new GCN architecture to combine information from different layers together so that we can utilize various hierarchical features and meanwhile make the GCN scheme faster. With the SGNet-101 as backbone and new GCN architecture, a new model named SGGCN is proposed by us.

## 2. Related Work

With the development of deep learning, researchers have achieved great performance in image classification tasks and made good efforts in medical image classification and segmentation. In the chest disease recognition task, the diseases share co-occurrence features and have hierarchical structures, so special techniques should be adopted to tackle this hierarchical multilabel learning classification task. ChestX-ray14 dataset [10] and CheXpert [11] dataset with hierarchical multilabel features have been widely used, as well as some methods with probability modelling, attention learning, and graph neural network are also introduced to learn the hierarchical features. Chen et al. [12] mainly focused on probability modelling and tried to predict the conditional probability for each label and fined-tuning this model with unconditional probability. Guan and Huang [13] used ResNet-50 or DenseNet-121 as the backbone, designed an attention module to obtain normalized attention scores, and integrated the features from backbone and the attention scores into a residual attention block to make classifications. In order to utilize the co-occurrence features in the datasets MS-COCO [14] and VOC2007, Chen and Wei et al. [8] used graph convolution network to capture the correlations of the labels and applied these features on the features extracted from input images by ResNet-101. Chen and Li et al. [15] further applied this graph convolution network method on multilabel cheset X-ray image classification and proposed CheXGCN, which achieved considerable results on Chest X-ray14 and CheXpert.

## 3. Methods

### 3.1. Word Embedding

GloVe [16] word embedding is adopted to convert label words into vectors so that this vector can take the place of the one-hot encoding. Our method used 300-dim word vectors from GloVe text model which trained on the Wikipedia dataset to convert the labels in the CheXpert dataset into vectors so that it produced a 14 × 300 matrix, and this matrix would further be fed into graph convolution network, which is regarded as Graph Convolution Network Module (GCNM) in SGGCN that we proposed.

### 3.2. Unbalanced Learning

As will be mentioned in Section 5.1, CheXpert datasets have unbalanced the data. The Fracture class have the least samples of 7270 with 484 uncertain, while the Lung Opacity has the largest samples of 92669 with 4341 uncertain. In order to tackle the imbalance of dataset, we adopted Weighted Cross Entropy Loss, which is proposed in CheXGCN:

(1) $$\begin{array}{c} L\left(p_{i},l_{i}\right)=-\omega_{p}\underset{l_{i}=1}{\sum }\log\left(\sigma \left(p_{i}\right)-\omega_{n}\underset{l_{i}=0}{\sum }\log\left(1-\sigma \left(p_{i}\right)\right)\right),\\ \omega_{p}=\frac{\left|P\right|+\left|N\right|+1}{\left|P\right|+1},\\ \omega_{n}=\frac{\left|P\right|+\left|N\right|+1}{\left|N\right|+1}, \end{array}$$

where *σ* is the sigmoid function and |*P*| and |*N*| are the number of positive samples and negative samples. In SGGCN, we computed |*P*| and |*N*| as the positive samples and negative samples in the whole training set to improve the stability.

### 3.3. Graph Neural Network

#### 3.3.1. Fourier Transform

When given a periodic function *f* (*x*), we can break it apart by Fourier series:

(2) $$\begin{array}{c} f\left(x\right)=\frac{\alpha_{0}}{2}\cdot 1+\overset{+\infty }{\underset{n=1}{\sum }}\alpha_{n}\sin\left(n\omega x\right)+\overset{+\infty }{\underset{n=1}{\sum }}b_{n}\cos\left(n\omega x\right),\\ a_{n}=\frac{\int_{0}^{T}f\left(x\right)\sin\left(n\omega x\right)\text{d}x}{\int_{0}^{T}\sin^{2}\left(n\omega x\right)\text{d}x},\\ b_{n}=\frac{\int_{0}^{T}f\left(x\right)\cos\left(n\omega x\right)\text{d}x}{\int_{0}^{T}\cos^{2}\left(n\omega x\right)\text{d}x}. \end{array}$$

It can be rewritten in a complex formula:

(3) $$\begin{array}{c} f\left(x\right)=\overset{+\infty }{\underset{n=-\infty }{\sum }}c_{n}e^{i}\frac{2\pi nx}{T}=\overset{+\infty }{\underset{t=-\infty }{\sum }}c_{t}e^{i\omega t}. \end{array}$$

It is noteworthy to mention that we can take {*e*^*iωt*^} as orthonormal set and take {*c*_*t*_} as the coordinate.

If we want to convert a nonperiodic function into Fourier series, we could regard it as a *T*=*∞* periodic function and use Fourier transform:

(4) $$\begin{array}{c} F_{T}\left(\omega \right)=\int_{-\infty }^{+\infty }f{\left(t\right)}^{-i\omega t}\text{dt}. \end{array}$$

When given *ω*, it used *e*^−*iωt*^ to decompose *f*(*t*) and get the coordinate of *e*^*iωt*^. And the inverse Fourier transform is

(5) $$\begin{array}{c} f\left(t\right)=\int_{-\infty }^{+\infty }F\left(w\right)e^{i\omega t}\text{dw}. \end{array}$$

#### 3.3.2. Graph Laplacian

When we consider Laplace operator in images, it can be defined by the sum of second derivative for the nearest four dimensions:

(6) $$\begin{array}{c} \Delta f=\overset{n}{\underset{i=1}{\sum }}\frac{\partial^{2}f}{\partial x_{i}^{2}}. \end{array}$$

If Laplace operator is moved into an undirected graph structure with *N* nodes, the Laplace operator of each node might be different due to the different relations and connections. The Laplace operator of node *i* should be defined as follows:

(7) $$\begin{array}{c} \Delta f_{i}=\underset{j}{\sum }\frac{\partial^{2}f}{\partial j^{2}}=\underset{j}{\sum }\omega_{ij}\left(f_{i}-f_{j}\right)\\ =\left(\underset{j}{\sum }\omega_{ij}f_{i}\right)-\underset{j}{\sum }\omega_{i}{\;}_{j}f_{j}\\ =d_{i}f_{i}-\omega_{i}f, \end{array}$$

where *f*_*i*_ is the function value of node *i*, *j* are the nodes connected with *i*, *ω*_*ij*_ is the weight of *i* − *j* connection, *d*_*i*_ is the degree of *i*, and *ω*_*i*_*f* is the sum of multiplication of all *j* and its weight. It can be rewritten in matrix form as follows:

(8) $$\begin{array}{c} \Delta f=\left(\begin{array}{ccc} d_{1} & \ldots & 0\\ \vdots & \ddots & \vdots \\ 0 & \cdots & d_{N} \end{array}\right)\left(\begin{array}{c} f_{1}\\ \vdots \\ f_{N} \end{array}\right)-\left(\begin{array}{c} -\omega_{i\cdot }-\\ \vdots \\ -\omega_{N\cdot }- \end{array}\right)\left(\begin{array}{c} f_{1}\\ \vdots \\ f_{N} \end{array}\right)\\ =\left(D-W\right)F=LF. \end{array}$$

And, we get the Laplacian matrix *L*, and we further get the normalized Laplacian matrix $\tilde{L}$.

(9) $$\begin{array}{c} \tilde{L}=D^{-1/2}\left(D-W\right)D^{-1/2}. \end{array}$$

The decomposition of Laplacian matrix *L* is

(10) $$\begin{array}{c} Lu_{k}=\lambda u_{k}. \end{array}$$

#### 3.3.3. Graph Fourier Transform

It can be proved by Helmholtz equation that *u*_*k*_ can be used as orthonormal set to decompose *f*_*i*_:

(11) $$\begin{array}{c} F_{k}\left(\lambda_{k}\right)={\hat{f}}_{k}\\ =\overset{N}{\underset{i=1}{\sum }}f_{i}u_{k}\left(i\right), \end{array}$$

where *λ*_*k*_ and *u*_*k*_ are the eigenvalues and eigenvectors of Laplacian matrix *L*, and *k*=1,…, *N* because *L* is an *N* × *N* symmetric matrix. It can be rewritten in matrix form:

(12) $$\begin{array}{c} \hat{f}=\left(\begin{array}{c} {\hat{f}}_{1}\\ \vdots \\ {\hat{f}}_{N} \end{array}\right)=\left(\begin{array}{ccc} u_{1}\left(1\right) & \ldots & u_{1}\left(n\right)\\ \vdots & \ddots & \vdots \\ u_{N}\left(1\right) & \cdots & u_{N}\left(N\right) \end{array}\right)\left(\begin{array}{c} f_{1}\\ \vdots \\ f_{N} \end{array}\right)\\ =U^{T}f. \end{array}$$

And, the inverse Fourier transform is

(13) $$\begin{array}{c} f=U\hat{f}. \end{array}$$

#### 3.3.4. Graph Convolution Network

According to convolution theorem, the Fourier transform of a convolution of two signals is the pointwise product of their Fourier Transforms under suitable conditions:

(14) $$\begin{array}{c} F\left\{f*g\right\}=F\left\{f\right\}\cdot F\left\{g\right\}, \end{array}$$

where *F* is the Fourier transform, *f* and *g* are two signals, *∗* is the convolution operation, and · is the pointwise product. When applied in graph *G*, with input *f* and kernel *h*, convolution operation in graph can convert to pointwise product under Fourier domain:

(15) $$\begin{array}{c} {\left(f*g\right)}_{G}=F^{-1}\left\{F\left\{f\right\}\cdot F\left\{h\right\}\right\}\\ =F^{-1}\left\{U^{T}f\cdot \hat{h}\right\}=U\left\{\left(\begin{array}{ccc} {\hat{h}}_{1} & \ldots & 0\\ \vdots & \ddots & \vdots \\ 0 & \cdots & h_{N}^{\wedge } \end{array}\right)U^{T}f\right\}\\ =U\left(\begin{array}{ccc} {\hat{h}}_{1} & \ldots & 0\\ \vdots & \ddots & \vdots \\ 0 & \cdots & h_{N}^{\wedge } \end{array}\right)U^{T}f=U\left(\begin{array}{ccc} \theta_{1} & \ldots & 0\\ \vdots & \ddots & \vdots \\ 0 & \cdots & \theta_{N} \end{array}\right)U^{T}f. \end{array}$$

The trainable variables *g* convert into *θ* in Fourier domain. And in graph neural network, we can directly learn *θ* instead of *g*. We also get the following formula, where *σ* is the activation function:

(16) $$\begin{array}{c} y=\sigma \left(U_{g_{\theta }}U^{T}x\right)\\ =\sigma \left(U\left(\begin{array}{ccc} \theta_{1} & \; & \;\\ \; & \ddots & \;\\ \; & \; & \theta_{N} \end{array}\right)U^{T}x\right). \end{array}$$

Here, we have defined the propagation rule of graph network. But this rule has some drawbacks: (1) *N* might be a large number, which would be due to large trainable parameters; (2) it is hard to share weight *θ*_*i*_ in *θ*; (3) *U* is computed from the decomposition of *L*, whose computation cost is *O*(*N*^3^). In order to tackle these problems, *g*_*θ*_ could be rewritten as a function *g*_*θ*_(·) in the following formula:

(17) $$\begin{array}{c} \left(\begin{array}{ccc} \theta_{1} & \; & \;\\ \; & \ddots & \;\\ \; & \; & \theta_{N} \end{array}\right)=g_{\theta }=g_{\theta }\left(\Lambda \right),\\ \Lambda =\left(\begin{array}{ccc} \lambda_{1} & \; & \;\\ \; & \ddots & \;\\ \; & \; & \lambda_{N} \end{array}\right). \end{array}$$

And Taylor series expansion is adopted to approximate *g*_*θ*_.

(18) $$\begin{array}{c} g_{\theta }\left(\Lambda \right)\approx \overset{K-1}{\underset{k=0}{\sum }}\theta_{k}\Lambda^{k}. \end{array}$$

This approximation takes the place of *g*_*θ*_(Λ), and we rewrite equation (16):

(19) $$\begin{array}{c} y=\sigma \left(U_{g_{\theta }}U^{T}x\right)=\sigma \left(U_{g_{\theta }}\left(\Lambda \right)U^{T}x\right)\\ \approx \sigma \left(U\left(\overset{K-1}{\underset{k=0}{\sum }}\theta_{k}\Lambda^{k}\right)U^{T}x\right)=\sigma \left(\overset{K-1}{\underset{k=0}{\sum }}\theta_{k}U\Lambda^{k}U^{T}x\right)\\ =\sigma \left(\overset{K-1}{\underset{k=0}{\sum }}\theta_{k}{\left(U\Lambda U^{T}\right)}^{k}x\right)=\sigma \left(\overset{K-1}{\underset{k=0}{\sum }}\theta_{k}L^{k}x\right). \end{array}$$

So here, we avoid the computation of decomposition of *L*, but *L*^*k*^ still suffers high computation cost. And Chebyshev polynomials are adopted to approximate *L*^*k*^:

(20) $$\begin{array}{c} L^{k}\approx T_{k}\left(\tilde{L}\right),\\ \tilde{L}=\frac{2}{\lambda_{\max}}L-I_{N},\\ T_{k}\left(L\right)=\left\{\begin{array}{cc} 1, & k=0,\\ L, & k=1,\\ 2LT_{K-1}\left(L\right)+T_{k-2}\left(L\right), & k\geq 2. \end{array}\right) \end{array}$$

And, equation (19) can be rewritten as follows:

(21) $$\begin{array}{c} y\approx \sigma \left(\overset{K-1}{\underset{k=0}{\sum }}\theta_{k}T_{k}\left(\tilde{L}\right)x\right). \end{array}$$

If *k* is set as 2, we get the following formula:

(22) $$\begin{array}{c} g_{\theta }*x\approx \overset{1}{\underset{k=0}{\sum }}\theta_{k}T_{k}\left(\tilde{L}\right)x\\ =\theta_{0}x+\theta_{1}\tilde{L}x. \end{array}$$

Since *θ*_0_ and *θ*_1_ influence the scale, it would be less effective after operation of normalization, so they can be set equal: *θ*=*θ*_0_=*θ*_1_, and equation (22) can be rewritten as follows:

(23) $$\begin{array}{c} g_{\theta }*x\approx \theta_{0}x+\theta_{1}\tilde{L}x\\ =\theta \left(I_{N}+\tilde{L}\right)x. \end{array}$$

And normalizing the matrix $A=I_{N}+\tilde{L}$, we get

(24) $$\begin{array}{c} A=I_{N}+\tilde{L},\\ A={\tilde{D}}^{-1/2}A{\tilde{D}}^{-1/2}. \end{array}$$

In order to learn the relations, weight *W* is introduced, and a new propagation rule can be obtained:

(25) $$\begin{array}{c} H^{\left(l+1\right)}=\sigma \left({\tilde{D}}^{-1/2}A{\tilde{D}}^{-1/2}H^{\left(l\right)}W^{\left(l\right)}\right), \end{array}$$

(26) $$\begin{array}{c} {\tilde{D}}_{ii}=\underset{j}{\sum }A_{ij}, \end{array}$$

(27) $$\begin{array}{c} A=I_{N}+\tilde{L}, \end{array}$$

(28) $$\begin{array}{c} \tilde{L}=\frac{2}{\lambda \max}L-I_{N}, \end{array}$$

where *H*^(*l*)^ is the output from layer *l* and *W*^(*l*)^ is the trainable variables in layer *l*. And the propagation rule in the graph convolution layer is

(29) $$\begin{array}{c} H^{\left(l+1\right)}=\sigma \left(\tilde{A}H^{\left(l\right)}W^{\left(l\right)}\right)\\ =\sigma \left({\tilde{D}}^{-1/2}A{\tilde{D}}^{-1/2}H^{\left(l\right)}W^{\left(l\right)}\right). \end{array}$$

### 3.4. Graph Presentation

In order to follow the propagation rule of equation (29), we should compute correlation matrix *A*. The way to compute *A* mentioned in equation (27) cannot work, because in this task, the graph is a weighted, directed graph.

We adopt the method introduced in ChexGCN, which used a nonlinear method to preprocess the correlation matrix *p* by equation (34) to reduce the noise and protect the correlations of labels:

(30) $$\begin{array}{c} A_{ij}=\left\{\begin{array}{cc} \lambda \frac{p_{ij}}{\sum_{i=0}^{C}P_{ij}+\theta }, & \text{if }P_{ij}\geq \phi ,\\ 0, & \text{if }P_{ij}<\phi , \end{array}\right) \end{array}$$

where *λ* is a hyperparameter to control the correlation state between the node and its neighborhood, *ϕ* is the threshold to filter the noise, and *θ* is an innately small quantity to ensure the denominator is not equal to zero.

## 4. Network Architecture

In this paper, we designed an efficient network architecture named SGGCN as illustrated in Figure 1, containing Feature Representation Module (FRM) and Graph Convolution Network Module (GCNM). The FRM used an SGNet-101 efficient neural network architecture to extract image features. GCNM used a small network architecture to extract correlations features from the labels. Finally, the features from FRM and GCNM are combined together and make multilabel prediction by matrix multiplication.

### 4.1. Feature Representation Module

In this module, we would use light models to extract image features with low computational consumption. Since some diseases like lung opacity have small scale and low resolution of feature maps might loss information of small target, especially pooling operation and convolution operation with large kernel scale would loss information. So, deep convolution neural network architectures like residual network can help to keep the information, but they suffer high computation cost. In order to design an efficient deep convolution neural network, ShuffleGhost Module is adopted to form ShuffleGhost Block and used this block to build a deep convolution neural network architecture SGNet-101. In ShuffleGhost Module, primary convolution conducts group convolution and generates primary feature with partial channels, and ghost convolution utilizes the redundant information of feature map to recover the ghost feature with rest channels by efficient operation like depthwise convolution; finally, the primary feature is concatenated with and ghost feature and disrupted the channel order with shuffle layer. So, ShuffleGhost can maintain the feature information with high computation efficiency, and SGNet-101 can extract features from multiple resolution with deep neural network.  Figure 2 shows the structure of ShuffleGhost Module and Block. One ShuffleGhost Block contains two ShuffleGhost Module; each one contains primary convolution part and ghost convolution part. In primary convolution part, group convolution is enrolled. In ghost convolution, cheap convolution is adopted to produce ghost feature map. The outputs from primary convolution part and ghost convolution part are concatenated together to generate output feature.

At the end of this module, the backbone SGNet-101 is followed by Global Average Pooling (GAP) layer to compress the features into 1024-d, where we denoted as *F*_FRM_.

### 4.2. Graph Convolutional Network Module

This module takes the embedding word of the labels and the graph presentation as input and uses graph convolution network to extract the correlation of the labels. The embedding words *X*_emb_ can be computed in Section 3.1, and the graph presentation $\tilde{A}$ is shown in equation (30). And *X*_emb_ and $\tilde{A}$ are fed to the first layer of IFE model:

(31) $$\begin{array}{c} H^{\left(1\right)}=\sigma \left(\tilde{A}X_{\text{emb}}W^{\left(0\right)}\right)\\ =\sigma \left(\tilde{A}H^{\left(0\right)}W^{\left(0\right)}\right), \end{array}$$

where *W*^(0)^ is the weight of the first layer, *H*^(1)^ is the output of the first layer, *σ* is the activation function, and *X*_emb_ is denoted as *H*^(0)^. The GCNM module consists of two graph convolution layers and one concatenate layer. For each graph convolution layers, the correlation information in different scale is extracted and generated as the output feature, and the output features from two graph convolution layers have the same shape as 512 × 14, and the two features are concatenated together to generate the output of GCNM module, which is denoted as matrix *W*. Finally, the information *F*_FRM_ and *W* from FRM and GCNM module are combined together by matrix multiplication, followed by sigmoid layer to generate multilabel class prediction.

## 5. Experiment

### 5.1. Datasets

This paper mainly focused on CheXPert datasets, which is widely used in deep hierarchical learning for chest disease recognition. The datasets have 14 classes (diseases); the label of each class is one of the four possible labels: NULL, −1, 0, and 1, and they represent empty, uncertain, negative, and positive, respectively. And the distribution of this dataset is illustrated as Table 1. We used CheXPert-v1.0-small (https://stanfordmlgroup.github.io/competitions/chexpert/) dataset, and the images in this dataset are not as high resolution as the origin CheXPert dataset, so this would influence the accuracy we can get in CheXGCN. The training set of this dataset has 223414 samples, and the label of each class might be one of four values as mentioned above. And the validation set has 234 samples, and the label of each class might be one of the two labels: positive and negative. After this procedure, the other NULL labels are replaced with negative labels.

At present, the testing dataset is not yet available, and some classes like Lung Leision, Plerual Other, and Fracture in the validation set are not enough. We divided the dataset into 70% for training, 10% for validation, and 20% for testing.

Table 1 is the summary of the training set. The right side is the summary of the validation set. The training set of this dataset has 223414 samples, and the label of each class might be one of four values as mentioned above. And the validation set has 234 samples, and the label of each class might be one of the two labels: positive and negative.

### 5.2. Hierarchical Labels

Since this paper focuses on hierarchical learning, this means that label *i* might have a strong relationship with label *j*. The label NULL does not simply mean negative, because in fact, if disease *i* is a subset of disease *j*, doctors do not need to check disease *j* if disease *i* is positive, so disease *j* is denoted by NULL.

In this situation, the disease *j* is positive if disease *i* is positive, although the label of disease *j* is NULL. If we replace NULL with negative, we would loss this relation and decrease the correlation between these two diseases. We notice that the validation set only has positive and negative labels in each class, which contain abundant information of relations among the classes. We use the validation set to mine the information.

The method this paper used is to compute the conditional probability for each pair of 14 diseases. When computing conditional probability of *i* when *j*: *P*(*i|j*), firstly, count the number *i* and *j* both appear in validation set *X*_*νa*_:

(32) $$\begin{array}{c} N\left(i,j\right)=\overset{N}{\underset{n=1}{\sum }}\pi \left(X_{va}\left(n,i\right)=1\right.,\left.X_{va}\left(n,j\right)=1\right), \end{array}$$

where *N* is the number of samples and *π* is the indicator function. Later, count the number *j* appear in *X*_*νa*_.

(33) $$\begin{array}{c} N\left(j\right)=\overset{N}{\underset{n=1}{\sum }}\pi \left(\left.X_{va}\left(n,j\right)=1\right)\right). \end{array}$$

And, it can be approximated *P*(*i|j*) as follows:

(34) $$\begin{array}{c} P\left(i|j\right)=\frac{N\left(i,j\right)}{N\left(j\right)+10^{-6}}. \end{array}$$

So, the conditional probability for each pair of 14 diseases can be computed. The result is illustrated in Table 2. It is noteworthy to mention that the probability *p* at row *j* and column *i* means *P*(*i|j*). We can find the following relations:

(35) $$\begin{array}{c} P\left(\text{Enca}=1|\text{Card}=1\right)=1, \end{array}$$

(36) $$\begin{array}{c} P\left(\text{Opca}=1|\text{Atel}=1\right)=1, \end{array}$$

(37) $$\begin{array}{c} P\left(\text{Opca}=1|\text{Pnuel}=1\right)=1, \end{array}$$

(38) $$\begin{array}{c} P\left(\text{Opac}=1|\text{Cons}=1\right)=1, \end{array}$$

(39) $$\begin{array}{c} P\left(\text{Opac}=1|\text{Edema}=1\right)=1, \end{array}$$

where Enca, Card, Opca, Atel, Pnue1, Cons, and Edema mean enlarged cardiomediastinum, atelectasis, pneumonia, consolidation, and edema. And, we do not take the positive labels in Lesi (lung lesion), Other (pleural other), and Frac (fracture) into consideration because of the lack of data. And, this paper mainly used the relations equations (35)–(38) because these relations can be proved medically. In this way, we can fill some NULL, Negative, and Uncertain labels in training set to positive labels if it meets the relations above.  Table 3 illustrates the result of the extended training data.

### 5.3. Model Training

In order to discuss the computation and accuracy performance of SGGCN we proposed, we would make comparison with models with backbones of ResNet-101 and MobileNetV2 [17] in Feature Representation Module, respectively. We set *θ*, *ϕ*, and *λ* to 10^−6^, 0.30, and 0.10 respectively, according to equation (30). In the exploratory experiment, we set initial learning rate *lr* to 10^−3^ and decent to 0.1 × *lr* every 5 epoch, as well as set the max epochs to 20, and trained SGGCN with scratch, GCN with ResNet-101 and MobileNetV2 with pretrained models. In order to discuss the performance of GCN, we also trained SGNet-101 without GCNM module.

### 5.4. Results

We trained SGGCN, GCN with ResNet-101 (denoted as ResNet-101-GCN), and MobileNetV2 (denoted as MobilenetV2-GCN), respectively, and get the performance on validation AUC trend as in Figure 3, and Table 4 illustrates the result of AUC on training, validation, and testing set, respectively. We could find that SGGCN-101 did not suffer from overfitting, and the performance on validation AUC and test AUC has about 3% lower than ResNet-101-GCN, where MobileNetV2-GCN has about 7% lower than ResNet-101-GCN.

Since the SGGCN-101, we focus on the efficient computing, and we compared the trainable parameters and FLOPs, as shown in Table 5. We could find SGGCN-101 and MobileNetV2-GCN meet a significant decrease in trainable parameters and FLOPs. When the trainable parameters and FLOPs meet about 80% decrease in SGGCN-101, it only has 3% decrease in validation AUC and test AUC.

### 5.5. Discussion

In graph convolution layers in GCNM in SGGCN, the weights are 300 × 512, 512 × 512, respectively. And as the structure of SGGCN in Figure 1, when the 14 × 300 embedding words are fed into GCNM, the features *H*^(1)^ and *H*^(2)^ from graph convolution layers are concatenated and form the output *W*_GCNM_, whose dimension is 14 × 1024. Then, *W*_GCNM_ is used to do matrix multiplication with the features extracted from FRM (Feature Representation Module). And we can find in this place that *W*_GCNM_ has similar action as a weight and carries attention information from GCNM module and weight the features in FRM. In order to discuss the influence of GCN, we trained SGNet-101 without GCNM module, which means that the model only has FRM module with backbone of SGNet-101 to extract features, but used a 14 × 1024 random initialed weight in the fully connected layer *W*_FC_ to do matrix multiplication with the features.

We used Principal Component Analysis [12] to do dimensionality reduction on both *W*_GCNM_ and *W*_FC_ and showed the result in Figure 4, where the first figure shows the PCA dimensionality reduction of *W*_GCNM_, as well as the second one shows that of *W*_FC_. We can find in the 2-dimensional subspace, the distances of these two classes Enlarged Cardiomediastinum and Cardiomegaly in both *W*_GCNM_ and *W*_FC_ are small, with 0.0862 of *W*_GCNM_ and 0.0410, and they all meet the rule of equation (35). But if we focus on the distances among these four diseases: Lung Opacity, Consolidation, Pneumonia, and Atelectasis, we can find *W*_GCNM_ works much better, because the mean distances among the four diseases is 0.2343, while the mean distances of *W*_FC_ is 0.3153. The first figure also shows that these four diseases are separated in the subspace of *W*_FC_, while the diseases in the subspace of *W*_GCNM_ still accumulated and retained relationships, and meet the rules of equations (36)–(38).

So far, we have found that *W*_GCNM_ can retain the information of equations (35)–(38), and we would mine more potential relationships information to explore its performance. Firstly, we extracted potential relationships information from training data by equation (34), and we got the conditional probability *P*(*i|j*). But in the result of dimensionality reduction, the way we judge the relationship of a pair classes is to compare their distance, which is an undirected information, while *P*(*i|j*) may be different from *P*(*i|j*) since it contains directed information. In order to tackle this problem, we compress the information of conditional probability into an undirected information:

(40) $$\begin{array}{c} I\left(i,j\right)=\frac{P\left(i|j\right)+P\left(j|i\right)}{2}. \end{array}$$

Table 6 shows the information matrix *I*. We consider using a threshold *ε* = 0.37 to find out the potential relationships of (*i*, *j*) pair if *I*(*i*, *j*) > *ε* and visualize them by adding edges onto Figure 4, and we get the result of Figure 5. We can find that except class Support Devices, *W*_GCNM_ also learn some potential relationships, which are not mentioned in equations (36)–(38), the distances of pairs (Edema, Lung Opacity), (Pleural Effusion, Lung Opacity), and (Pleural Effusion, Edema) are much smaller than those of *W*_FC_. Meanwhile, Lung Opacity has considerable relations with classes Pneumonia, Consolidation, Atelectasis, Edema, and Pleural Effusion, and it is placed in the center of them in the dimensionality reduction of *W*_GCNM_, while the dimensionality reduction of *W*_FC_ does not have those appearances.

We later applied dimensionality reduction on the outputs of 8000 samples in validation set from SGGCN and SGNet-101, respectively. In detail, we applied PCA on 14 classes, respectively, reduced the data to two dimensions, and applied Gaussian Mixture Model with one class to fit an analogous Gaussian distribution.  Figure 6 shows the dimensionality reduction of the output. The three figures in the first row show the 2D-PCA from the output of 14 classes, pair (Enlarged Cardiomediastinum, Cardiomegaly) and [Pleural Opacity, Consolidation, Pneumonia, Atelectasis] from SGGCN. And the second row shows the result from SGNet-101. We can find that although *W*_GCNM_ can take the correlation information, when conducting matrix multiplication with features from FRM, the appearance seems not considerable.

## 6. Conclusion

In this paper, an efficient X-ray classification method SGGCN is proposed, which adopts SGNet-101 backbone built with ShuffleGhost Module and applies this method on CheXpert datasets to do chest disease classification. We also compare the AUC, trainable parameters, and FLOPs with ResNet-101 with GCN and MobileNetV2 with GCN. It is found that although the trainable parameters and FLOPs meet a significant decrease, SGGCN still keeps a high AUC on validation and testing set.

## Figures and Tables

**Figure 1:** The architecture of SGGCN.

**Figure 2:** The structure of ShuffleGhost Block and Module.

**Figure 3:** The AUC performance trend on validation set of SGGCN-101, ResNet-101-GCN, and MobileNetV2-GCN.

**Figure 4:** PCA is adopted to reduce the data into two dimensions on both *W*_GCNM_ and *W*_FC_. The left figure is the PCA result of *W*_GCNM_; the other is that of *W*_FC_.

**Figure 5:** The undirected information matrix *I* when set threshold *ε*=0.37.

**Figure 6:** The first row shows the 2D-PCA from the output of 14 classes.

**Table 1:** Summary of 14 classes in CheXPert dataset (https://stanfordmlgroup.github.io/competitions/chexpert/).

Pathology	Positive	Negative	Uncertain	Empty	Pathology	Positive	Negative
No finding	22381	0	0	201033	No finding	38	196
Enlarged cardiom.	10798	21638	12403	178575	Enlarged cardiom.	109	125
Cardiomegaly	27000	11116	8087	177211	Cardiomegaly	68	166
Lung opacity	105581	6599	5598	105636	Lung opacity	126	108
Lung lesion	9186	1270	1488	211470	Lung lesion	1	233
Edema	52246	20726	12984	137458	Edema	45	189
Consolidation	14783	28097	27742	152792	Consolidation	33	201
Pneumonia	6039	2799	18770	195806	Pneumonia	8	226
Atelectasis	33376	1328	33739	154971	Atelectasis	80	154
Pneumothorax	19448	56341	3145	144480	Pneumothorax	8	226
Pleural effusion	86187	35396	11628	90203	Pleural effusion	67	167
Pleural other	3523	316	2653	216922	Pleural other	1	233
Fracture	9040	2512	642	211220	Fracture	0	234
Support devices	116001	6137	1079	100197	Support devices	107	127

**Table 2:** The condition probability of 14 classes in CheXpert.

	Nofi	Enca	Card	Opac	Lesi	Edem	Cons	Pnue1	Atel	Pneu2	Effu	Other	Frac	Devi
Nofi	1	0	0	0	0	0	0	0	0	0	0	0	0	0
EnCa	0	1	0.624	0.752	0.009	0.339	0.220	0.037	0.477	0.028	0.431	0	0	0.495
Card	0	1	1	0.765	0	0.324	0.265	0.059	0.515	0.015	0.441	0	0	0.515
Opac	0	0.651	0.413	1	0.008	0.357	0.262	0.063	0.635	0.048	0.476	0.008	0	0.492
Lesi	0	1	0	1	1	0	0	0	1	0	0	0	0	1
Edem	0	0.822	0.489	1	0	1	0.311	0.044	0.467	0.022	0.356	0	0	0.533
Cons	0	0.727	0.545	1	0	0.424	1	0.242	0.818	0.030	0.818	0.030	0	0.485
Pneu1	0	0.500	0.500	1	0	0.250	1	1	0.875	0	0.875	0.125	0	0.375
Atel	0	0.650	0.437	1	0.012	0.262	0.337	0.087	1	0.012	0.612	0.012	0	0.525
Pneu2	0	0.375	0.125	0.750	0	0.125	0.125	0	0.125	1	0.250	0	0	0.500
Effu	0	0.701	0.448	0.896	0	0.239	0.403	0.104	0.731	0.030	1	0.015	0	0.493
Other	0	0	0	1	0	0	1	1	1	0	1	1	0	1
Frac	0	0	0	0	0	0	0	0	0	0	0	0	0	0
Devi	0	0.505	0.327	0.579	0.009	0.224	0.150	0.028	0.393	0.037	0.308	0.009	0	1

**Table 3:** The summary of some classes that are extended by proposed method.

	Pathology	Positive	Negative	Uncertain	Empty
Origin	Enlarged cardiom.	10798	21638	12403	178575
Proposal	Enlarged cardiom.	35897	21466	12092	153959
Origin	Lung opacity	105581	6599	5598	105636
Proposal	Lung opacity	134262	6081	3984	79087

**Table 4:** The AUC performance on the result of AUC on training, validation, and testing set of SGGCN-101, ResNet-101-GCN, and MobileNetV2-GCN.

Models	Train AUC	Valid AUC	Test AUC
ResNet-101-GCN	0.8528	0.8075	0.8080
SGGCN-101	0.8027 (−5.87%)	0.7834 (−2.98%)	0.7831 (−3.08%)
MobileNetV2-GCN	0.7650 (−10.30%)	0.7509 (−7.01%)	0.7531 (−6.79%)

**Table 5:** The trainable parameters and FLOPs of ResNet-101-GCN, SGGCN-101, and MobileNetV2-GCN.

Structure	Trainable parameters	FLOPs
ResNet-101-GCN	47,308,864	16,017,450,516
SGGCN-101	12,427,684 (−73.73%)	3,072,345,732 (−80.82%)
MobileNetV2-GCN	5,459,712 (−88.46%)	661,395,120 (−95.88%)

**Table 6:** The undirected information matrix *I*.

	Nofi	Enca	Card	Opac	Lesi	Edem	Cons	Pnue1	Atel	Pneu2	Effu	Other	Frac	Devi
Nofi	1	0	0	0	0	0	0	0	0	0	0	0	0	0.233
EnCa	0	1	0.875	0.379	0.072	0.315	0.090	0.060	0.149	0.058	0.297	0.074	0.098	0.369
Card	0	0.875	1	0.361	0.045	0.329	0.073	0.050	0.127	0.034	0.287	0.049	0.061	0.358
Opac	0	0.379	0.361	1	0.354	0.466	0.555	0.522	0.624	0.333	0.627	0.325	0.272	0.621
Lesi	0	0.072	0.045	0.354	1	0.057	0.066	0.065	0.070	0.068	0.195	0.056	0.038	0.185
Edem	0	0.315	0.329	0.466	0.057	1	0.137	0.113	0.217	0.052	0.407	0.048	0.064	0.465
Conso	0	0.090	0.073	0.555	0.066	0.137	1	0.118	0.100	0.045	0.291	0.052	0.036	0.298
Pneu1	0	0.060	0.050	0.522	0.065	0.113	0.118	1	0.059	0.015	0.153	0.028	0.019	0.155
Atel	0	0.149	0.127	0.624	0.070	0.217	0.100	0.059	1	0.126	0.339	0.061	0.088	0.388
Pneu2	0	0.058	0.034	0.333	0.068	0.052	0.045	0.015	0.126	1	0.209	0.041	0.084	0.350
Effu	0	0.297	0.287	0.627	0.195	0.407	0.291	0.153	0.339	0.209	1	0.133	0.150	0.534
Other	0	0.074	0.049	0.325	0.056	0.048	0.052	0.028	0.061	0.041	0.133	1	0.063	0.193
Frac	0	0.098	0.061	0.272	0.038	0.064	0.036	0.019	0.088	0.084	0.150	0.063	1	0.215
Devi	0.233	0.369	0.358	0.621	0.185	0.465	0.298	0.155	0.388	0.350	0.534	0.193	0.215	1

## Data Availability

The datasets used and/or analyzed during the current study are available from the corresponding author upon reasonable request.
